This article has been retracted.

# Application of Meditation Relaxation Training and Rosenthal Effect in Patients with Adenoidectomy

**DOI:** 10.1155/2022/1420639

**Published:** 2022-09-26

**Authors:** Wei Jun, Yue Tian

**Affiliations:** Otorhinolaryngology Head and Neck Surgery Department, The Second Affiliated Hospital of Harbin Medical University, No. 246, Xuefu Road, Nangang District, Harbin, Heilongjiang 150001, China

## Abstract

**Objective:**

This study aims to explore the application effect of meditation relaxation training and the Rosenthal effect in patients with adenoidectomy.

**Methods:**

This study included 94 children who underwent adenoidectomy in our hospital from April 2020 to May 2022 and were divided into a study group and a control group. The control group was given routine care, and the study group was given meditation relaxation training and the Rosenthal effect on the basis of the control group. The negative emotions, treatment compliance, complication rates, and nursing satisfaction of children's family members before and after the intervention were compared between the two groups.

**Results:**

The results of this study showed that after the intervention, the CDI and SCARED scores of the children in the study group were significantly lower than those in the control group. The treatment compliance in the study group was significantly higher than that in the control group, and the incidence of complications was significantly lower than that in the control group.

**Conclusion:**

The intervention of meditation relaxation training and the Rosenthal effect on children with adenoidectomy can relieve their negative emotions, improve treatment compliance, reduce the incidence of complications, and the children's family members are more satisfied.

## 1. Introduction

Adenoid hypertrophy is a common disease in children, mainly, inflammation of the nasopharynx and adjacent parts, as well as pathological hyperplasia caused by repeated stimulation of adenoids by adenoid autoinflammation, including pharyngeal discomfort, nasal obstruction, snoring, mouth breathing, nasal congestion, and other symptoms [1, 2]. Conventional conservative treatment of adenoid hypertrophy can alleviate the disease, but it is difficult to completely eradicate the lesions, which may easily lead to repeated attacks. Adenoidectomy is an important minimally invasive treatment for this disease, with the advantages of fewer traumas, less blood loss, and faster postoperative recovery. However, children with adenoid hypertrophy are younger and prone to nervousness and fear during treatment, resulting in poor treatment compliance and unfavorable surgical treatment [3, 4]. Therefore, it is highly important to provide effective nursing intervention during adenoidectomy treatment [5].

Routine care only focuses on disease treatment and lacks sufficient attention to the patient's psychological state, resulting in poor results [6]. Meditation relaxation training is an open self-conscious attention process, which is an important clinical psychological intervention. It is simple to operate, easy to master, and is of great significance for regulating physical and mental states [7]. The Rosenthal effect is also an important clinical intervention model, mainly through positive psychological cues such as praise, trust, and expectation to improve individual self-esteem and self-confidence, change their behavior habits, and encourage them to face treatment positively [8].

This study aimed to select 94 children with adenoidectomy in our hospital to explore the combined intervention value of meditation relaxation training and Rosenthal effect in groups, in order to provide new ideas for the clinical intervention of the disease.

## 2. Materials and Methods

### 2.1. General Information

A total of 94 children with adenoidectomy in our hospital from April 2020 to May 2022 were enrolled in this study. The inclusion criteria for this study were the following. (1) All patients underwent adenoidectomy under general anesthesia in our hospital. (2) The child's family members have good communication skills. The exclusion criteria for this study were (1) those with organic lesions of the kidney, liver, heart, and other organs. (2) Those with language communication impairment and cognitive dysfunction. (3) Those with congenital deformities. (4) Patients who underwent oral and laryngeal surgery 6 months before enrollment. According to the simple random number table method, patients were divided into the study and the control groups, with 47 cases in each. There were 26 males and 21 females in the study group; age 5–10 years, mean (6.54 ± 1.19) years; disease duration 0.5–4.5 years, mean (2.51 ± 1.37) years; body mass index 18.3–24.5 kg/m^2^, average (21.39 ± 3.02) kg/m^2^. In the control group, there were 29 males and 18 females; age 5–10 years, mean (6.29 ± 1.24) years; disease duration 0.5–5 years, mean (2.63 ± 1.51) years; and body mass index 18.1–24.8 kg/m^2^, average (21.56 ± 2.96) kg/m^2^. The clinical data of the two groups were balanced and comparable (*P* > 0.05). The study protocol was approved by the ethics committee of the second affiliated hospital of Harbin Medical University. All family members of patients signed the informed consent forms.

### 2.2. Treatment

The patients in the control group were given daily nursing care and assisted in the preoperative examination. One day before the operation, the operation process, anesthesia method, postoperative discomfort symptoms, and corresponding treatment methods were introduced. Within 2 hours after the operation, local cold compresses or ice cubes containing sodium chloride were used for analgesia, and atomization treatment was carried out in strict accordance with the doctor's instructions to relieve postoperative pain. Instruct patients to eat cold liquid food 4–6 hours after surgery, and encourage patients to exercise independently with the assistance of medical staff or family members.

On the basis of the control group, the patients in the study group used meditation relaxation training and the Rosenthal effect. Soundproof doors and windows and carpets were placed in the ward to reduce noise, and health posters related to sample excision were posted prominently in the ward. Actively communicate with patients and their families. Through the psychological intervention of nurses, we guide patients to accept their own disease and recovery process and help patients establish healthy and positive recovery behaviors through self-motivation and positive psychological suggestions. Reasonably match negative emotions and better emotional states, subtly changed the physical and mental states of patients with poor emotional states and reduced their fears and other psychology. Timely assess the patient's condition and physical and mental state during the intervention period, discuss the corresponding treatment measures immediately after discovering the problem and optimize the nursing intervention plan. Before relaxation, meditation relaxation training first guides the patient to choose the meditation object. In the first stage, the body is relaxed for 5 minutes to ensure the quietness of the ward, assist the patient to lie supine, and effectively relax the muscles. In the second stage, adjust the breathing for 5 minutes, guide the patient to self-regulate breathing according to the instructions, breathe slowly, and feel the feeling of the gas passing through the nasal cavity and oral cavity. At this stage, you need to pay attention to the patient's breathing frequency. After adjusting the breathing several times, guide the patient to adjust the breathing rate. Focus on what happened before the meditation. The patient is then instructed to close his eyes slightly and visualize himself in the picture, while guiding the patient's fantasy to extend the picture.

### 2.3. Observation Indicators

Negative emotions before and after the interventions in the two groups were counted. According to the evaluation of the Children's Self-rating Depression Inventory (CDI) and the Screening Scale for Children's Anxiety and Mood Disorders (SCARED), the total score of the CDI was 54 points, and the total score of SCARED was 82 points. High depression and anxiety are more intense. The treatment compliance of the two groups was counted, and the self-made treatment compliance scale (after the pretest, the internal consistency reliability of this scale was 0.93, and the validity coefficient was 0.91) to evaluate, with a total of 10 points. 9–10 points for complete compliance, 7-8 points for partial compliance, less than 7 points for noncompliance, treatment compliance = (complete compliance + partial compliance)/total number of cases × 100%. The incidence of complications in the two groups was calculated. The nursing satisfaction of the families of the children in the two groups was calculated, and the Newcastle Nursing Satisfaction Scale (NSNS) was used to evaluate the scores, which were divided into very satisfied, satisfied, generally satisfied, dissatisfied, and very dissatisfied. Total satisfaction = (very satisfied + satisfied)/total number of cases × 100%.

### 2.4. Statistical Analysis

The data were analyzed by SPSS 22.0 (IBM SPSS Statistics, USA). The measurement data were presented as mean ± standard deviation (SD). The differences were determined by the two-sided unpaired Student's *t*-test. *P* < 0.05 was considered statistically significant.

## 3. Results

### 3.1. Negative Emotions

As shown in Table 1, before the intervention, there were no significant differences in the CDI (42.89 ± 5.07 vs. 41.56 ± 6.11) and SCARED (69.54 ± 8.16 vs. 67.24 ± 9.05) points between the study and control groups (*P* > 0.05). After the intervention, the scores of CDI (21.65 ± 3.77) and SCARED (33.08 ± 3.38) in the study group were significantly lower than those in the control group (CDI: 27.11 ± 4.54 and SCARED: 38.34 ± 4.62) (*P* < 0.05).

### 3.2. Treatment Compliance

As shown in Table 2, the treatment compliance in the study group (93.62%) was significantly higher than that in the control group (78.72%) (*P* < 0.05).

### 3.3. Complication Rate

As shown in Table 3, the incidence of complications in the study group (2.13%) was significantly lower than that in the control group (17.02%) (*P* < 0.05).

### 3.4. Nursing Satisfaction of Children's Family Members

The nursing satisfaction of the families of children in the study group (95.74%) was significantly higher than that in the control group (82.98%) (*P* < 0.05, Table 4).

## 4. Discussion

Adenoid hypertrophy can lead to insufficient lung expansion and poor breathing in children. In severe cases, it can cause thoracic deformity and abnormal growth hormone secretion, which will affect growth and development to varying degrees [9]. Adenoidectomy is an important measure in the clinical treatment of adenoid hypertrophy. With the aid of endoscopy, lesions can be effectively removed and clinical symptoms can be improved. However, due to the patient's young age, fear of surgery, and poor compliance with treatment, it will affect the smooth progress of surgery and increase the risk of complications [10, 11]. Therefore, it is of great significance to take effective nursing measures to intervene in pediatric adenoidectomy.

Routine nursing measures are mainly based on disease observation, surgical cooperation, and explanation of relevant precautions, which are difficult to meet the comprehensive needs of patients, and the overall effect, is difficult to achieve an ideal state [12]. Meditation and relaxation training is an important clinical intervention. It is mainly a self-regulation method in which individuals consciously maintain their attention on the current external/internal experience without any evaluation. It can effectively downregulate the key hormone cortisol content in stress response. Relief from a negative emotional state can also improve the individual's ability to regulate emotions to a certain extent. In addition, the individual is in a state of physical and mental relaxation during the intervention period, which is conducive to helping the individual effectively cope with and deal with related negative emotions [13–15]. The Rosenthal effect is also a commonly used clinical psychological adjustment measure. It is also known as the “expectation effect”. It mainly improves individual behavior through motivation, praise, trust, and expectation. It is a new nursing model. Expectation-action-acceptance in the process of internalization, positive psychological hints are given by affirmation and encouragement, to achieve the purpose of adjusting the physical and mental state [16].

There are no clinical reports on the specific application value of meditation relaxation training and the Rosenthal effect in pediatric adenoidectomy. The results of this study showed that after the intervention, the CDI and SCARED scores of the children in the study group were significantly lower than those in the control group. The treatment compliance in the study group was significantly higher than that in the control group, and the incidence of complications was significantly lower than that in the control group. It is feasible and effective for children with adenoidectomy to be combined with the aerial effect to help relieve their negative emotional state and encourage them to accept adenoidectomy with a positive attitude so as to ensure the effectiveness and safety of surgical treatment and reduce the incidence of complications. The main reasons are as follows; the meditation relaxation training can increase the activity of the left prefrontal brain area and strengthen positive emotions. At the same time, the amygdala is the initiation area of negative emotions, and the medial prefrontal lobe layer is driven by the amygdala. The bridge of bad emotions, through meditation and relaxation training, one can affect the corresponding areas of the dorsal medial/lateral prefrontal cortex to play a role in stress response inhibition and cultivate their inner attention to the current, not subjectively judge emotional changes and perceptions, and truthfully accept the current reality [17–20]. The Rosenthal effect attaches great importance to children's psychological feelings, focusing on relieving children's negative emotional state and reducing psychological stress through anticipation, trust, praise, and encouragement, which is conducive to children's active venting of negative emotions and reducing physical and mental burden, and the dried cranberry exercises taken during the intervention period can adjust the individual's cognition of their own diseases and treatment through the power of mindfulness, avoid falling into blind psychological troubles, and prevent excessive psychological reactions.

In addition, from the results of this study, it can also be known that the nursing satisfaction of the children in the study group (95.74%) was higher than that in the control group (82.98%) after the intervention (*P* < 0.05), indicating that the meditation relaxation training combined with the Rosenthal effect intervention mode is also effective. To a certain extent, it can deepen the recognition of the clinical work by the families of children with adenoidectomy, which is of great significance to reducing disputes between nurses and patients and establishing the image of high-quality nursing services in the hospital. The physical and mental state of the patient can encourage him to actively cooperate with the treatment, thereby reducing the risk of complications, improving the effectiveness and safety of the treatment, relieving his clinical symptoms, and shortening the recovery process of the child, so the family members of the child are more satisfied.

To sum up, the intervention of meditation relaxation training and the Rosenthal effect on children with adenoidectomy can relieve their negative emotions, improve treatment compliance, reduce the incidence of complications, and improve the children's family satisfaction.

## Figures and Tables

**Table 1:** Comparison of negative emotion scores between the two groups (min).

Time	Group	Number of cases	CDI	SCARED
*Before intervention*	Study	47	42.89 ± 5.07	69.54 ± 8.16
	Control	47	41.56 ± 6.11	67.24 ± 9.05
	*t* value		1.148	1.294
	*P* value		0.254	0.199

*After intervention*	Study	47	21.65 ± 3.77	33.08 ± 3.38
	Control	47	27.11 ± 4.54	38.34 ± 4.62
	*t* value		6.343	6.299
	*P* value		<0.001	<0.001

**Table 2:** Comparison of treatment compliance between the two groups (%).

Group	Number of cases	Full compliance	Partial compliance	Non-compliance	Treatment compliance
Study	47	29 (61.70)	15 (31.91)	3 (6.38)	44 (93.62)
Control	47	21 (44.68)	16 (34.04)	10 (21.28)	37 (78.72)
*χ* ^2^ value					4.374
*P* value					0.036

**Table 3:** Comparison of the incidence of complications between the two groups (%).

Group	Number of cases	Nasal bleeding	Adenoid residual hyperplasia	Infection	Total incidence
Study	47	1 (2.13)	0 (0.00)	0 (0.00)	1 (2.13)
Control	47	3 (6.38)	2 (4.26)	1 (2.13)	8 (17.02)
*χ* ^2^ value					4.424
*P* value					0.035

**Table 4:** Comparison of nursing satisfaction of family members of the two groups of children (%).

Group	Number of cases	Very satisfied	Satisfied	Generally satisfied	Dissatisfied	Very dissatisfied	Total satisfaction
Study	47	33 (70.21)	12 (25.53)	1 (2.13)	1 (2.13)	0 (0.00)	45 (95.74)
Control	47	26 (55.32)	13 (27.66)	4 (8.51)	3 (6.38)	1 (2.13)	39 (82.98)
*χ* ^2^ value							4.029
*P* value							0.045

## Data Availability

All data are included within the article.
